The article "Baseline Plasma Gas6 Protein Elevation Predicts Adverse Outcomes in Hospitalized COVID-19 Patients" was published in 2022. Journal: Dis Markers.

# Baseline Plasma Gas6 Protein Elevation Predicts Adverse Outcomes in Hospitalized COVID-19 Patients

**DOI:** 10.1155/2022/1568352

**Published:** 2022-04-29

**Authors:** Stelvio Tonello, Manuela Rizzi, Erica Matino, Martina Costanzo, Giuseppe Francesco Casciaro, Alessandro Croce, Eleonora Rizzi, Erika Zecca, Anita Pedrinelli, Veronica Vassia, Raffaella Landi, Mattia Bellan, Luigi Mario Castello, Rosalba Minisini, Venkata Ramana Mallela, Davide D'Onghia, Gian Carlo Avanzi, Mario Pirisi, Daniele Lilleri, Pier Paolo Sainaghi

**Affiliations:** ^1^Department of Translational Medicine, Università del Piemonte Orientale (UPO), Novara 28100, Italy; ^2^CAAD, Center for Autoimmune and Allergic Diseases, Università del Piemonte Orientale (UPO), Novara, Italy; ^3^Rheumatology Unit, AOU “Maggiore della Carità”, Novara 28100, Italy; ^4^Department of Internal Medicine and COVID-19 Unit, AOU “Maggiore della Carità”, Novara 28100, Italy; ^5^Division of Emergency Medicine and COVID-19 Sub-Intensive Unit, AOU “Maggiore della Carità”, Novara 28100, Italy; ^6^Division of Internal Medicine, Azienda Ospedaliera “SS. Antonio e Biagio e Cesare Arrigo”, Alessandria 15100, Italy; ^7^Unit of Microbiology and Virology, IRCCS Policlinico San Matteo Foundation, Pavia 27100, Italy

## Abstract

Reliable biomarkers allowing early patients' stratification for the risk of adverse outcomes in COVID-19 are lacking. Gas6, together with its tyrosine kinase receptors named TAM, is involved in the regulation of immune homeostasis, fibrosis, and thrombosis. Our aim was to evaluate whether Gas6, sAxl, and sMerTK could represent early predictors of disease evolution either towards a negative (death or need of ICU admission) or a positive (discharge and/or clinical resolution within the first 14 days of hospitalization) outcome. To this purpose, between January and May 2021 (corresponding to third pandemic wave in Italy), 139 consecutive SARS-CoV-2 positive patients were enrolled in a prospective observational study. Plasma levels of these molecules were measured by ELISA at the time of hospitalization and after 7 and 14 days. We observed that higher plasma Gas6 concentrations at hospital admission were associated with a worsening in clinical conditions while lower sMerTK concentrations at baseline and after 7 days of hospitalization were associated with a more favorable outcome. At multivariate analysis, after correction for demographic and COVID-19 severity variables (NEWS2 and PiO_2_/FiO_2_), only Gas6 measured at baseline predicted an adverse prognosis with an odds ratio of 1.03 (C.I. 1.01-10.5). At ROC curve analysis, baseline Gas6 levels higher than 58.0 ng/ml predicted a severe disease evolution with 53.3% sensitivity and 77.6% specificity (area under the curve 0.653, *p* = 0.01, likelihood ratio of 2.38, IQR: 1.46-3.87). Taken together, these results support the hypothesis that a dysregulation in the Gas6/TAM axis could play a relevant role in modulating the course of COVID-19 and suggest that plasma Gas6 may represent a promising prognostic laboratory parameter for this condition.

The article "Baseline Plasma Gas6 Protein Elevation Predicts Adverse Outcomes in Hospitalized COVID-19 Patients" was published in 2022. Journal: Dis Markers.

## 1. Introduction

Since the end of 2019, the world is facing a novel severe acute respiratory syndrome, named COVID-19 [1–3]. The causative agent of COVID-19 is a positive single-stranded RNA virus named SARS-CoV-2, a *β*-coronavirus which displays genetic similarities with two other coronavirus, SARS-CoV and MERS-CoV, responsible for two other severe pneumonia outbreaks in 2002 and 2012, respectively [1, 4, 5].

COVID-19 displays a wide range of clinical manifestations, from a nearly asymptomatic condition to a severe interstitial pneumonia with respiratory failure requiring hospitalization burdened with a high mortality rate [5–7] in particular in high risk population [5, 8].

In patients experiencing the most severe COVID-19 clinical manifestations, a hyperinflammatory response is often observed, also defined as cytokine storm syndrome, together to a prothrombotic condition, multiorgan failure, and high risk of death [4, 9–12].

Gas6 (growth arrest specific gene 6) is a 75 kDa secreted glycoprotein expressed by many human cells and tissues (i.e., heart, lungs, stomach, kidney, gut, pancreas, bone, and endothelium). It is a vitamin K-dependent protein involved in many biological processes, such as cell proliferation, adhesion, and migration, as well as phagocytosis and apoptosis regulation. Moreover, it is also known to be involved in the control of inflammatory responses and platelet function, as well as in modulating fibrotic evolution after chronic inflammation [13–18].

In order to exert its biological functions, Gas6 needs to interact with a specific tyrosine kinase receptor family, named TAM, consisting of 3 different receptors (Tyro-3, Axl, and MerTK). All the 3 TAM receptors can be isolated in human plasma as soluble decoy receptors (sTAM, namely, sTyro-3, sAxl, and sMerTK) deriving from proteolytic cleavage of the membrane receptor mediated by ADAM10 and ADAM17 metalloproteinases [13, 14, 17, 19–21].

TAM receptors are differentially expressed in the human body, with only Axl showing a diffuse expression. Upon ligand binding, TAM receptors become activated and mediate several cellular responses, such as stimulation of cell growth, inhibition of apoptosis, stimulation of hemostasis, and modulation of inflammation and immune responses [17, 21, 22].

The article "Baseline Plasma Gas6 Protein Elevation Predicts Adverse Outcomes in Hospitalized COVID-19 Patients" was published in 2022. Journal: Dis Markers.

It is known that Gas6 binds with the strongest affinity to Axl and to a lesser extent to Tyro3 and MerTK: while acting as immune regulator, the Gas6 activation finally results in dampening Toll-like receptors inflammatory signaling [13, 19, 20, 22, 23] thus counteracting inflammatory responses induced also by pathogen infections [9, 20]. Consistently, in a recent study, performed during the first wave of COVID-19 pandemic, Morales and coworkers [9] evaluated plasma Gas6 and TAM receptors expression in a Spanish cohort of COVID-19 patients, highlighting that Gas6 levels measured at admission in an emergency care unit were directly correlated to disease severity. Similar results were obtained during the same period of time (first wave of the pandemic, spring 2020) also by other independent research groups [24, 25], showing an interesting correlation between Gas6 levels and disease outcome.

In this paper, we aim to analyze plasma Gas6, sAxl, and sMerTK levels in a prospective cohort of hospitalized SARS-CoV-2 positive patients that underwent standard therapy (corticosteroids and heparin) to evaluate if Gas6 and/or TAM levels measured at hospital admission and during hospitalization may predict COVID-19 in-hospital trajectory as well as treatment response.

## 2. Patients and Methods

### 2.1. Patients

We performed a prospective cohort observational study including 139 consecutive patients admitted to nonintensive care unit (ICU) wards (including high dependency/subintensive units) of “Maggiore della Carità” University Hospital in Novara (Italy) between January and May 2021 (during the third Italian pandemic wave). These patients are part of a larger multicentric observational study cohort (BIAS (Baseline Immunity status effect on sArs-cov2 presentation and evolution: comparison between immunocompetent and immunocompromised patientS) study). The study protocol was approved by the local ethical committee (CE 7/21) and was conducted in strict accordance with the Declaration of Helsinki. Patients giving their informed consent to the enrollment were included if they were adults (>18 years), SARS-CoV-2 positive (assessed by molecular RT-PCR or antigenic test), with clinical symptoms not exceeding 12 days. Exclusion criteria were defined as follow: severe clinical presentation suggestive of an imminent death or requiring an immediate ICU admission, advanced oncological condition (i.e., not suitable for medical or surgical treatment), and stage V renal failure.

All patients included received a standard of care treatment, according to the “Maggiore della Carità” Hospital internal protocol for the management of COVID-19 (oxygen supplementation, corticosteroids, and low molecular weight heparin (LMWH) unless contraindicated).

The article "Baseline Plasma Gas6 Protein Elevation Predicts Adverse Outcomes in Hospitalized COVID-19 Patients" was published in 2022. Journal: Dis Markers.

### 2.2. Endpoint Definition

The endpoint definition is as follows: (1) identification of plasma Gas6 and sTAM receptors (sAxl and sMerTK) values predicting, at baseline and after 7 days of hospitalization, a negative outcome (in-hospital death or ICU admission); (2) identification of plasma Gas6 and sTAM receptors (sAxl and sMerTK) values predicting, at baseline and after 7 days of hospitalization, a rapid clinical recovery (discharge and/or National Early Warning Score (NEWS2) ≤ 2 for at least 24 hours within the first 14 days of hospitalization).

### 2.3. Blood Sample Collection

Blood samples for Gas6, sAxl and sMerTK quantifications were collected by venous puncture using EDTA as anticoagulant at different time points during hospitalization (at baseline (t0) and after 7 and 14 days of hospitalization (t7 and t14)). Blood fractions were immediately separated by centrifugation and stored at -80°C until the time of analysis.

### 2.4. Soluble Axl Quantification

sAxl levels were determined by ELISA technique using a commercial kit (R&D Systems DuoSet Elisa DY154, McKinley, MN, USA) following the manufacturer instructions. Prior to sAxl quantification, plasma samples were diluted 1 : 50 [9] in dilution reagent (provided by the manufacturer). Absorbance was recorded using a Victor X4 microplate reader (Perkin Elmer, Waltham, MA, USA). Optical density at 450 nm was fitted versus a calibration curve prepared with Axl standard (0 ng/ml-4 ng/ml range) by applying a four-parameter logistic regression as suggested by the manufacturer.

### 2.5. Soluble MerTK Quantification

sMerTK levels were determined by ELISA technique using a commercial kit (R&D Systems DuoSet Elisa DY6488, McKinley, MN, USA) following the manufacturer instructions. Prior to sMerTK quantification, plasma samples were diluted 1 : 10 [9] in dilution reagent (provided by the manufacturer). Absorbance was recorded using a Victor X4 microplate reader (Perkin Elmer, Waltham, MA, USA). Optical density at 450 nm was fitted versus a calibration curve prepared with MerTK standard (0 ng/ml-4 ng/ml range) by applying a four-parameter logistic regression as suggested by the manufacturer.

### 2.6. Gas6 Quantification

Plasmatic Gas6 levels were determined by ELISA technique according to Alciato and coworkers' protocol [26] validated and used for Gas6 quantification in several human diseases and in different body fluids [13, 22, 27–29]. Prior to Gas6 quantification, plasma samples were diluted 1 : 50 [9] in PBS. Absorbance was recorded using a Victor X4 microplate reader (Perkin Elmer, Waltham, MA, USA). Optical density at 450 nm was fitted versus a calibration curve prepared with Gas6 standard (0 ng/ml-2 ng/ml range) by applying a four-parameter logistic regression.

The article "Baseline Plasma Gas6 Protein Elevation Predicts Adverse Outcomes in Hospitalized COVID-19 Patients" was published in 2022. Journal: Dis Markers.

### 2.7. Data Collection and Statistical Analysis

Relevant data of each patient (demographics, clinical parameters, therapeutic schedule, laboratory parameters) were stored and managed on a web-based database (RedCap platform). Clinical and laboratory data were collected by carefully reviewing medical records, starting from the time of hospital admission (baseline, t0) until discharge (or for a maximum of 28 days) or study exit (death or ICU admission). Data extracted from RedCap database and Gas6, sAxl, and sMerTK quantifications underwent statistical analysis to evaluate their significance toward the expected endpoints. For continuous variables, the measures of central tendency and dispersion were medians and interquartile range (IQR). Categorical variables were presented as frequency (percentage). Variables were compared with the Mann–Whitney *U* test (continuous variables) or Pearson *χ*^2^ test (categorical variables). Statistically significant biomarkers identified in the univariate analysis were used to build multivariable logistic regression models. ROC curves were built to identify the prognostic cut-off for the parameters of interest. The threshold chosen to indicate statistical significance was 0.05 (two-tailed). Statistical analyses were performed with Statistica for Windows release 12 (TIBCO Software Inc., Palo Alto, CA, USA) and MedCalc® Statistical Software version 20.014 (MedCalc Software Ltd., Ostend, Belgium).

## 3. Results

We enrolled and followed prospectively 139 SARS-CoV-2 positive patients (86 males (61.9%), median age 63.8 years (IQR: 56.2-71.9 years)) admitted to non-ICU wards of “Maggiore della Carità” Hospital in Novara (Italy). Baseline population characteristics were already described in a precedent study [30]. Briefly, at admission, 118 patients (80.6%) showed a moderate to severe (PiO_2_/FiO_2_ < 200) respiratory failure. Patient severity was also confirmed by the median NEWS2 score of 5 (IQR: 4-6) assessed at the time of hospital admission. Dyspnea and dry cough were the most common symptoms at hospital admission (62.6% and 38.9%, respectively). Noteworthy, when hospitalized, 83 of the 139 selected patients were already on COVID-19-related home treatment (corticosteroids (52.5%), azithromycin (35.2%), heparin (30.9%), and 69.9% received these drugs in combination).

Among the 139 patients meeting the inclusion criteria for the study, 29 died during hospitalization or were transferred to ICU. Out of the remaining 110 patients, 91 were discharged or reached a NEWS2 ≤ 2 for at least 24 hours within the first 14 days of hospitalization.

The article "Baseline Plasma Gas6 Protein Elevation Predicts Adverse Outcomes in Hospitalized COVID-19 Patients" was published in 2022. Journal: Dis Markers.

Plasma Gas6, sAxl, and sMerTK concentrations were evaluated at baseline (t0) and at different time points (t7 and t14) during hospital stay (Table 1).

We then compared median plasma Gas6, sAxl, and sMerTK concentrations observed in patients with an unfavorable in-hospital outcome (deceased or transferred to ICU) with those of all other patients. As evident in Table 2, baseline plasma Gas6 concentration was significantly increased among subjects who had an adverse outcome thereafter.

Plasma Gas6, sAxl, and sMerTK concentrations were then compared between those patients who had a faster recovery from COVID-19 pneumonia (hospital discharge or NEWS2 ≤ 2 for at least 24 hours within 14 days of hospitalization) and all the other patients. Plasma sMerTK concentration resulted to be significantly lower either at baseline or at 7 days of hospitalization in patients with a faster recovery (Table 3).

At a multivariate analysis, baseline plasma Gas6 concentration retained its prognostic role after correction for demographic (age and gender) and disease severity-related (NEWS2 score and PiO_2_/FiO_2_) variables at baseline as evidenced in Table 4.

On the other hand, sMerTK concentration, either at baseline or at 7 days of hospitalization, lost its prognostic role after correction for demographic (age and gender) and disease severity-related (NEWS2 score and PiO_2_/FiO_2_) variables (multivariable analysis models: sex (female) *β* 0.0828, *p* = 0.3165, odds ratio 0.26, 95% CI 0.09-0.76; age *β* -0.3437, *p* = 0.0001, odds ratio 1.06, 95% CI 1.02-1.11; NEWS2 *β* 0.0616, *p* = 0.4372, odds ratio 0.89, 95% CI 0.70-1.11; PiO_2_/FiO_2_*β* 0.1978, *p* = 0.0177, odds ratio 0.99, 95% CI 0.99-1.00; sMerTk t0 *β* -0.0767, *p* = 0.3374, odds ratio 1.00, 95% CI 0.97-1.04. Sex (female) *β* -0.02612, *p* = 0.8082, odds ratio 0.32, 95% CI 0.07-1.53; age *β* -0.3895, *p* = 0.0006, odds ratio 1.10, 95% CI 1.03-1.18; NEWS2 *β* 0.0067, *p* = 0.94952, odds ratio 0.89 95% CI 0.64-1.26; PiO_2_/FiO_2_*β* -0.0098, *p* = 0.9929, odds ratio 1.00, 95% CI 0.99-1.02; sMerTk t7 *β* -0.1646, *p* = 0.1355, odds ratio 1.03, 95% CI 0.97-1.10).

According to the results presented above, we built ROC curve for baseline plasma Gas6 to predict an adverse prognosis.  Figure 1 shows the ROC curve referred to baseline Gas6 levels: considering an area under the curve of 0.653, we identified a Gas6 level of 58.0 ng/ml as the cut-off predicting a more severe disease evolution (53.33% sensitivity and 77.57% specificity), with a likelihood ratio of 2.38 (IQR: 1.46-3.87).

## 4. Discussion

In this observational prospective cohort study about patients affected by moderate to severe COVID-19 pneumonia in an acute care hospital setting, we observed that baseline plasma Gas6 concentration is higher in patients with an adverse outcome while sMerTK at baseline and at 7 days from hospitalization is lower in patients with a quicker resolution of the disease (discharged from hospital or NEWS2 ≤ 2 within 14 days) even if the results about sMerTK were not confirmed after correction for demographic and disease severity variables. Moreover, a specific cut-off for plasma Gas6 concentration at the baseline had a good accuracy in predicting an adverse prognosis.

The article "Baseline Plasma Gas6 Protein Elevation Predicts Adverse Outcomes in Hospitalized COVID-19 Patients" was published in 2022. Journal: Dis Markers.

The finding that Gas6 plasmatic levels correlate with COVID-19 severity is not surprising from the pathophysiologic point of view. In fact, Gas6 is involved in inflammatory conditions [9, 17, 21] and plays a role in thrombosis pathophysiology [31, 32] and in fibrosis evolution triggered by chronic inflammation [20]. The higher Gas6 levels observed in patients developing a more severe illness may be related to the degree of activation of the innate immunity response that is responsible for the hyperinflammation observed in these patients [9, 33]. Moreover, the Gas6/TAM axis also plays a pivotal role in assuring vessel wall homeostasis and in regulating platelet activation in response to vascular damage [15, 22, 32]. Since the alveolar damage in COVID-19 is associated to vessel injury with diffuse thrombotic activation, the observed dysregulation in Gas6/TAM pathway can be associated also to these events as a link between inflamed and damaged endothelium and platelet activation. Moreover, the Gas6/TAM axis is also known to regulate fibrotic response triggered by chronic inflammation in many clinical conditions, such as liver cirrhosis and pulmonary fibrosis [20, 22]. It is known that pulmonary fibrosis can be a threatening COVID-19 complication, affecting at least one-third of hospitalized patients [34–36]. Consistently, the dysregulation in Gas6/TAM physiological balance with the elevation of Gas6 at baseline in patients with the most severe prognosis may be associated to an increased acute/subacute fibrosis evolution responsible for the irreversible or hardly reversible respiratory failure seen in the most severe COVID-19 cases.

In a recent work, it has been observed that plasma Gas6 levels measured at emergency ward were a prognostic marker of disease severity in the Spanish cohort enrolled during the first pandemic wave [9]. Even if our study confirms Morales and coworkers' [9] observation on Gas6 prognostic role, it is noteworthy that the two cohorts are significantly different. Morales and colleagues enrolled their patients in a short period of time during the first Spanish wave of the pandemic (27-31 March 2020), while we enrolled our patients during the third Italian wave (January–May 2021). Such difference in the timing of enrollment accounts for a wide difference both in disease severity at admission and in the hospital management. In Morales and coworkers' study, patients were enrolled among unselected patients admitted to the emergency ward with different disease severity, including milder cases, while the majority of the patients included in our study had moderate to severe respiratory failure, as confirmed by NEWS2 score and PiO_2_/FiO_2_ values at the time of hospital admission, therefore burdened with a worse prognosis. Additionally, while during the first wave of the pandemic, there were no standardized therapeutic protocols available to treat severe COVID-19 manifestations; nowadays, there are some evidence-based guidelines supporting the use of corticosteroids and heparin to treat hospitalized SARS-CoV-2 positive patients [37–42]. As a further confirmation of the differences existing between ours and the Spanish cohort, no information about the pharmacological treatment was available for Morales and coworkers' study, while in our study, all the SARS-CoV-2 positive patients during their hospital stay received a standardized therapy based on corticosteroids (dexamethasone or methylprednisolone) and low molecular weight heparin. Results in accordance with those of Morales and colleagues were obtained also by De Bruin and coworkers [24], who screened 64 biomarkers potentially linked to COVID-19 disease evolution in two different populations (COVID-19 positive patients admitted to general and ICU wards), showing a correlation between Gas6 dynamic changes in patients admitted to ICU and subsequent death. Likewise, these two cohorts appeared to be different from ours: as Morales and coworkers did, also De Bruin's group enrolled patients during the first wave of COVID-19 pandemic; moreover, these patients were treated according to the Amsterdam UMC internal protocol that included thromboprophylaxis but not corticosteroids or other immunomodulatory agents. Furthermore, Huckriede and colleagues [25] studied Gas6 in severe, ICU admitted, COVID-19 patients, observing lower levels of this cytokine in survivors compared to nonsurvivors. Also, this cohort has relevant differences compared to ours: again, patients were enrolled during the first wave of the pandemic only on ICU-admitted subjects, of which only few underwent steroid-based therapy.

The article "Baseline Plasma Gas6 Protein Elevation Predicts Adverse Outcomes in Hospitalized COVID-19 Patients" was published in 2022. Journal: Dis Markers.

Concerning Gas6 levels, our results are not only a simple confirmation of these previous data but add a more precise context where plasma Gas6 measurement is worthwhile: the patients with COVID-19 needing hospitalization due to moderate to severe respiratory failure needing noninvasive ventilation.

Moreover, in our study, Gas6 plasmatic levels were evaluated not only at the baseline but also at different time points during hospital stay, showing a decrease over time, even if not statistically significant. Such results thus confirm the assumption that Gas6 behaves as an acute phase biomolecule [43, 44], possibly involved in both the hyperinflammatory and the prothrombotic and hypercoagulable state observed in severe COVID-19 [45, 46].

It is known that Gas6, to carry out its biological functions, needs to interact with specific receptors: for this reason, in our study, we also evaluated two sTAM receptors, namely, sAxl and sMerTK. Both these receptors are detectable in plasma after proteolytic cleavage of the membrane bound form by disintregrins ADAM10 and ADAM17, one of the regulation mechanisms that our organism use to modulate their activity [13, 14, 17, 19–21].

In our study, we did not find any statistically significant difference in sAxl levels, while we observed lower sMerTK levels both at the baseline and after 7 days of hospitalization in patients with a more favorable disease evolution (i.e., discharge and/or NEWS2 ≤ 2 within 14 days of hospitalization). Even if not confirmed at multivariate analysis, our data on sMerTK levels are in partial accordance with those of Morales and coworkers' [9] where higher baseline sMerTK values were associated to the worsening of clinical conditions in COVID-19 patients.

Altogether, our results highlighted the involvement of Gas6/TAM system in COVID-19 evolution, in particular when hyperinflammation and immune response dysregulation is present. Consistently, Gas6 may represent an early response mechanism to limit viral infection damages and subsequent cytokine storm [9, 19]. Moreover, our results evidenced that Gas6 measured at hospital admission may represent a useful biomarker to stratify risk of hospitalized patients to adverse evolution. Such early stratification may assist clinicians in identifying those patients who will benefit of a higher intensity of care setting or of an early anticytokine treatment.

We are aware that this study may have several limitations. First of all, it was focused on hospitalized COVID-19 patients, referring moderate or severe disease symptoms, so it is not possible to extend our results to all those patients with mild symptoms or even asymptomatic. Another limitation is based on the mono-centric nature of this study and limited numerosity: patient enrollment was performed at a single hospital center, so that a prospective multicentric validation of the obtained results is needed to recommend Gas6 measurement in clinical practice. Furthermore, this study was performed in clinical practice, so that slight differences in patients' treatment may have occurred; however, all patients were treated according to our hospital treatment protocol guiding corticosteroids and heparin regimens, thus limiting relevant differences. Finally, in the statistical analysis, we assumed a linear behavior of our data, so that it is possible that some confounding factors could have influenced the obtained results.

The article "Baseline Plasma Gas6 Protein Elevation Predicts Adverse Outcomes in Hospitalized COVID-19 Patients" was published in 2022. Journal: Dis Markers.

## 5. Conclusions

In this prospective observational cohort study, we evidenced that a higher plasma Gas6 concentration at hospital admission predicted a more severe evolution in patients affected by moderate to severe COVID-19 pneumonia. So that, plasma Gas6 measurement at the baseline might represent a promising biomarker in COVID-19 to help to stratify patients' severity. Additionally, we confirmed that Gas6/TAM system is involved in COVID-19 with severe evolution and may be a promising target for further research on COVID-19 pathophysiology.

## Figures and Tables

**Figure 1:** ROC curve for Gas6 plasmatic levels at the time of hospital admission predicting a severe disease evolution.

**Table 1:** Plasma Gas6, sAxl, and sMerTK concentrations at different time points (t0, t7, and t14). Values are expressed as median (IQR).

Laboratory findings (ng/ml)	Median (IQR)
*Gas6*	
t0	46.8 (38.2-59.6)
t7	36.6 (27.7-45.9)
t14	36.1 (28.1-41.7)
sAxl	
t0	16.7 (10.7-27.4)
t7	26.2 (14.9-39.6)
t14	22.5 (15.7-29.8)
*sMerTK*	
t0	33.7 (25.3-38.4)
t7	28.0 (21.4-34.8)
t14	24.3 (21.2-30.3)

**Table 2:** Comparison of plasma Gas6, sAxl, and sMerTK concentrations at different time points (t0, t7, and t14) between patients with an adverse disease evolution (deceased or transferred to ICU) vs. all other patients. Values are expressed as median (IQR). Bold text highlights the statistically significant results.

Laboratory findings (ng/ml)	Adverse disease evolution (*n* = 29)	All other patients (*n* = 110)	*Z*	*p* value
**Gas6**				
t0	**58.3 (43.8-75.2)**	**46.0 (37.3-57.9)**	**-2.548**	**0.011**
t7	40.5 (36.9-45.5)	34.6 (26.9-47.0)	-1.552	0.121
t14	38.3 (28.6-86.2)	36.1 (28.1-41.4)	-0.580	0.562
**sAxl**				
t0	18.8 (9.5-26.7)	16.0 (10.7-27.8)	-0.057	0.954
t7	33.3 (14.7-49.2)	25.8 (15.1-39.4)	-0.496	0.620
t14	20.3 (17.8-32.3)	23.1 (14.8-29.8)	-0.433	0.665
**sMerTK**				
t0	36.9 (21.8-39.6)	33.2 (26.5-38.2)	-1.148	0.251
t7	31.5 (21.9-33.7)	26.9 (21.4-35.2)	-0.939	0.348
t14	21.2 (20.9-21.3)	25.3 (21.9-34.2)	1.530	0.126

**Table 3:** Comparison of plasma Gas6, sAxl, and sMerTK concentrations at different time points (t0, t7, and t14) between patients with a faster recovery (discharged from hospital and/or NEWS2 ≤ 2 within 14 days) and all the other patients. Values are expressed as median (IQR). Bold text highlights the statistically significant results.

Laboratory findings (ng/ml)	Faster clinical recovery (*n* = 91)	All other patients (*n* = 48)	*Z*	*p* value
**Gas6**				
t0	46.44 (38.8-58.0)	48.9 (36.8-67.6)	-1.116	0.264
t7	32.5 (26.9-47.0)	39.9 (33.7-45.9)	-1.201	0.230
t14	29.7 (23.6-41.1)	36.8 (32.9-51.2)	-1.683	0.092
**sAxl**				
t0	16.9 (11.8-28.5)	15.9 (9.7-22.4)	0.992	0.321
t7	26.4 (15.9-45.0)	24.1 (10.7-35.2)	1.241	0.214
t14	23.3 (17.4-29.8)	20.3 (15.2-32.3)	0.066	0.947
**sMerTK**				
t0	**32.3 (25.5-37.0)**	**37.0 (25.3-41.4)**	**-2.135**	**0.033**
t7	**26.6 (20.1-31.7)**	**32.6 (22.1-38.3)**	**-2.015**	**0.044**
t14	24.6 (20.6-32.5)	24.1 (21.2-28.1)	-0.022	0.982

The article "Baseline Plasma Gas6 Protein Elevation Predicts Adverse Outcomes in Hospitalized COVID-19 Patients" was published in 2022. Journal: Dis Markers.

**Table 4:** Multivariable analysis of plasma Gas6 concentration at baseline predicting an adverse disease evolution (death/ICU admission) including demographic and COVID-19 severity-related variables. Bold text highlights the statistically significant results.

Predictors (t0)	*β* ^∗^	*p* value	Odds ratio	95% confidence interval
Age	**0.2583**	**0.0022**	**1.07**	**1.02-1.12**
Sex (female)	**-0.2174**	**0.0102**	**0.24**	**0.08-0.723**
Gas6	**0.2084**	**0.0120**	**1.03**	**1.01-1.05**
PiO_2_/FiO_2_	-0.1260	0.1300	0.99	0.98-1.00
NEWS2	0.0456	0.5775	0.94	0.74-1.20

## Data Availability

Data are available upon reasonable request to be addressed to the corresponding author.
